The article "Neural Function Recovery and Safety of Mild Hypothermia Therapy Combined with Monosialotetrahexosylganglioside on Neonatal Asphyxia Complicated by Hypoxic Ischemic Encephalopathy" was retracted in 2023. Reasons: unreliable results or conclusions; concerns about the data; concerns about the peer review; concerns about the citations.

# Neural Function Recovery and Safety of Mild Hypothermia Therapy Combined with Monosialotetrahexosylganglioside on Neonatal Asphyxia Complicated by Hypoxic Ischemic Encephalopathy

**DOI:** 10.1155/2021/6186011

**Published:** 2021-12-27

**Authors:** Jingjing Ge, Xiaoling Jiao, Fanlin Qi, Hui Li

**Affiliations:** Department of Pediatrics, The Affiliated Yantai Yuhuangding Hospital of Qingdao University, Yantai 264001, Shandong Province, China

## Abstract

**Objective:**

To explore the effect and safety of mild hypothermia therapy combined with monosialotetrahexosylganglioside (GM1) on neural function recovery of neonatal asphyxia complicated by hypoxic ischemic encephalopathy (HIE).

**Methods:**

The clinical data of 90 neonates with HIE were retrospectively analyzed. According to the treatment methods, the neonates were divided into a routine group, a mild hypothermia group, and a combination group, with 30 cases in each group. The differences in neural function recovery, biochemical indexes, clinical signs recovery, efficacy, and complications were observed in the three groups after treatment.

**Results:**

After treatment, the score of neonatal behavioral neurological assessment (NBNA) and level of superoxide dismutase (SOD) in the combination group were higher than those of the other two groups (*P* < 0.05). The levels of neuron-specific enolase (NSE), S-100*β* protein, and plasma neuropeptide Y (NPY) in the combination group were lower than those in the other two groups, and the recovery time of consciousness, muscle tension, and reflex was shorter (*P* < 0.05). The combination group showed higher total effective rate and lower incidence of complications as compared with the other two groups (*P* < 0.05).

**Conclusion:**

Mild hypothermia therapy combined with GM1 for the treatment of neonatal asphyxia complicated by HIE can promote the recovery of neural function and reduce the incidence of complications in neonates.

## 1. Introduction

Neonatal hypoxic ischemic encephalopathy (HIE) is a common perinatal disease in clinic, which is mainly caused by perinatal asphyxia. In China, the incidence of HIE is increasing annually, which poses a serious threat to the life safety of neonates [1]. Even if the neonates survive, they may still suffer from severe neural dysfunction, which not only affects the development of intelligence but undoubtedly increases the socioeconomic and medical burden [2]. In view of this, it is urgent to find an effective therapeutic method for HIE.

At present, the pathogenesis of HIE has not yet been fully clarified [3], while the previous treatment schemes lack specificity [4, 5]. In recent years, mild hypothermia therapy has been shown to be effective in treating HIE and reducing the mortality of affected neonates [6, 7]. However, this treatment has certain requirements for the onset time window of children and may also cause a series of adverse reactions such as fat necrosis and arrhythmia in neonates [8]. With the emergence of a new type of brain injury drug, monosialotetrahexosylganglioside (GM1), the treatment for HIE has entered a new era. GM1 plays a positive role in the growth, differentiation, and regeneration of neurons [9] and has been widely used in the treatment of acute ischemic stroke, Alzheimer's disease, and other cerebrovascular diseases [10, 11]. A study has shown that GM1 used in HIE treatment can improve the short-term clinical efficacy and reduce long-term neurodevelopmental disorders in neonates [12]. In addition, GM1 combined with hyperbaric oxygen therapy for HIE can effectively improve the short- and long-term nervous system development in neonates [13]. Moreover, GM1 combined with mild hypothermia therapy can better promote the recovery of neural function and improve clinical symptoms in neonates with HIE. Currently, the research on the treatment of HIE with mild hypothermia combined with GM1 has become a hot spot of clinical concern. It has been proved that mild hypothermia therapy combined with GM1 can reduce convulsions, promote recovery of consciousness, and protect nerve function in neonates with HIE. But research on the mechanism of action and safety of this combined therapy is still insufficient, which warrants large-scale clinical studies for confirmation. Based on existing research, this study is aimed at further exploring the effects and safety of hypothermia therapy combined with GM1 on neurological recovery of neonatal asphyxia complicated by HIE.

## 2. Materials and Methods

### 2.1. General Data and Grouping

This is a retrospective study which was reviewed and approved by the Ethics Committee of Yan Tai Yu Huang-ding Hospital. The clinical data of 90 neonates with HIE admitted to our hospital from May 2020 to May 2021 were analyzed. The included newborns were divided into routine group, mild hypothermia group, and combined group according to the treatment method, with 30 cases in each group. The guardians of the included subjects were fully informed of the contents and purpose of this study and signed the informed consent.

Inclusion criteria are as follows: (1) complete clinical data; (2) in accordance with the diagnostic criteria of HIE [14]; (3) gestational age > 36 weeks and birth weight > 2000 g; (4) a history of intrapartum asphyxia or intrauterine distress during childbirth, with spontaneous breathing after rescue for over 10 minutes; (5) coma, abnormal nerve reflexes, and convulsions within 6 hours of birth while without obvious abnormalities in electroencephalography; and (6) time from onset to treatment < 6 hours.

Exclusion criteria are as follows: (1) severe congenital malformations or structural dysfunction of the heart or other vital organs, (2) severe infection, (3) family refusal to cooperate during treatment, and (4) death within 28 days after delivery.

### 2.2. Data Collection and Research Methods

#### 2.2.1. Data Collection

The general data of neonates were collected, including the gestational age, day age, sex, birth weight, Apgar score at 5 minutes after birth (5 m Apgar), asphyxia score, and neural function [15]. Since the degree of neonatal asphyxia may be misdiagnosed by using 5 m Apgar alone, the asphyxia score was also used to further determine the degree of neonatal asphyxia and the comparability among the 3 groups before intervention.

#### 2.2.2. Research Methods

Neonates in the routine group received routine treatment measures [16]. (1) Oxygen inhalation and assisted ventilation were given to stabilize the internal environment. (2) Interventions were given against convulsions. Intracerebral activators were used to reduce intracranial pressure and relieve cerebral edema. (3) Stable circulation capacity and balance of water and electrolyte were maintained. (4) Symptomatic treatments were given. The treatment lasted for 10 days.

Neonates in the mild hypothermia group were treated with mild hypothermia therapy on the basis of the routine group. Six hours after birth, the neonate was placed naked on a hypothermia pad, the head was cooled with a medical temperature controller (RC-2000, Jilin Richeng, China), and the cooling cap was adjusted in an automatic mode. The rectal temperature was measured once every 10 minutes to reach the temperature of 33-34°C within 1 hour. After 72 hours, the neonates were allowed to rewarm naturally or assisted rewarming if the rewarming was not ideal. The course of treatment was 10 days.

On the basis of the mild hypothermia group, the combination group was additionally given GM1 injection (Qilu Pharmaceutical, China, H20046213) 20 mg/day, once a day for 10 days.

#### 2.2.3. Outcome Measures

Primary outcome measures included the neural function as well as plasma superoxide dismutase (SOD), plasma neuropeptide Y (NPY), serum S-100*β* protein, and serum neuron-specific enolase (NSE) levels.

Secondary outcome measures were treatment efficiency and complications.

#### 2.2.4. Evaluation Methods for Outcome Measures

The HIE scale included 3 degrees, mild, moderate, and severe [17]. Mild was indicated when the neonate was irritable, with normal muscle tension, normal or easily induced hug reflex, and no convulsions. Moderate was considered when the neonate was lethargic or inhibited, with low muscle tension, weakened sucking reflex and hug reflex, and convulsions. Severe was translated in coma, extremely low muscle tension, areflexia, unequal pupils, frequent or persistent seizures, irregular breathing, apnea, or respiratory failure.

The heart rate, respiration, muscle tension, laryngeal reflex, and skin color of the neonates 5 minutes after birth were scored by the 5 m Apgar score. Each item was assigned 0-2 points, with a total score of 10 points. A score of 8-10 points indicated normal condition, 4-7 points indicated mild asphyxia, and 0-3 points indicated severe asphyxia.

Based on the preliminary screening with 5 m Apgar score, the degree of asphyxia was further assessed from respiration, heart rate, skin color, blood oxygen saturation, partial pressure of oxygen, partial pressure of carbon dioxide, arterial cord blood pH, and noninvasive blood pressure. Each item was assigned 0-2 points, with a total score of 18 points. A score less or equal to 6 points was considered as severe asphyxia, 7-10 points as mild asphyxia, and over 11 points as normal. The neurological function of the three groups was evaluated on admission and the next day after the completion of treatment, and the levels of plasma SOD, plasma NPY, serum S-100*β*, and serum NSE were determined in the next early morning after admission and the next morning after the end of treatment.

The neurological function of neonates was evaluated using the neonatal behavioral neurological assessment (NBNA) from 5 aspects of behavioral ability, passive muscle tension, active muscle tension, primitive reflex, and general assessment, with a total score of 40 points. A score less than 35 points indicated neurological abnormalities in neonates.

Enzyme-linked immunosorbent assay (ELISA) was used to detect the levels of plasma SOD, plasma NPY, serum S-100*β*, and serum NSE in neonates. The kits used were human SOD ELISA kit, human NPY ELISA kit, human S-100*β* ELISA kit, and human NSE ELISA kit all purchased from Shanghai EK-Bioscience Biotechnology Co., Ltd. (Cat. Nos. EK-H11804, EK-H11491, EK-H12486, and EK-H11495).The experimental procedures were carried out strictly in accordance with the kit instructions.

Efficacy was evaluated based on daily observation and recording of the neonate's vital signs, consciousness, basic reflexes, and muscle tension, as well as NBNA scores evaluated on the 7th day of treatment. Markedly effective was translated in stable vital signs, basically restored consciousness, reflexes and muscle tensions, and a NBNA score ≥ 38 points. Effective corresponded to alleviated clinical symptoms, improved observation indicators, and a NBNA score of 36-38 points. No improvement or aggravation in conditions and a NBNA score of less than 36 points was considered as ineffective. Effective rate = (cases of markedly effective + cases of effective)/total number of cases∗100%.

#### 2.2.5. Statistical Methods

The SPSS 25.0 software was used to statistically process the data. Count data, which were expressed as number of cases and percentage (*n*, %), were analyzed using the *χ*^2^ test. Measurement data were expressed in the form of mean ± standard deviation (*x̅*±sd). Independent sample *t* test was used for intergroup comparisons, paired-samples *t* test was used for intragroup comparisons before and after treatment, and one-way ANOVA was used for pairwise comparisons. *P* < 0.05 was considered statistically significant.

## 3. Results

### 3.1. Comparison of General Data

There was no significant difference in sex, gestational age (week), day age, birth weight, degree of asphyxia, 5 m Apgar score, and HIE severity among the three groups (*P* > 0.05) (Table 1).

### 3.2. Comparison of Neural Function among the Three Groups before and after Treatment

There was no significant difference in the NBNA score among the three groups upon admission (*P* > 0.05). After treatment, the NBNA score increased in all the three groups (*P* < 0.05). The score was the highest in the combination group, followed in descending order by the mild hypothermia group and the routine group (*P* < 0.05) (Table 2 and Figure 1).

### 3.3. Comparison of SOD, NPY, S-100*β*, and NSE Levels among the Three Groups before and after Treatment

SOD, NPY, S-100*β*, and NSE levels are all associated with the neurological damage or repair process in children with HIE. Therefore, detection of these four indicators is helpful to identify the changes of neurological function in HIE. There was no difference in the levels of SOD, NPY, S-100*β*, and NSE among the three groups on admission (*P* > 0.05). After treatment, the level of SOD increased while the levels of NPY, S-100*β*, and NSE decreased in all the three groups (*P* < 0.05). The increase in SOD and the decreases in NPY, S-100*β*, and NSE were the most significant in the combination group, and those in the mild hypothermia group were more significant compared with the routine group (*P* < 0.05) (Table 3 and Figures 2(a)–2(d)).

### 3.4. Comparison of the Recovery of Clinical Signs among the Three Groups during Treatment

During treatment, the recovery time of clinical signs in terms of consciousness, reflex, and muscle tension was the shortest in the combination group, and the recovery time of clinical signs in the mild hypothermia group was significantly lower than that in the routine group (*P* < 0.05) (Table 4 and Figure 3).

### 3.5. Comparison of Efficacy among the Three Groups

After treatment, the total effective rate was the highest in the combination group, followed in descending order by the mild hypothermia group and the routine group (*P* < 0.05) (Table 5).

### 3.6. Comparison of Complications among the Three Groups during Treatment

During treatment, the number of cases of epilepsy, cerebral palsy, and respiratory failure in the combination group was lower than that in the other two groups, and the difference in the incidence of total complications was statistically significant among the three groups (*P* < 0.05) (Table 6).

## 4. Discussion

HIE seriously threatens the life and health of neonates and affects the long-term intellectual development of neonates [18]. Mild hypothermia therapy has been proven to be an effective treatment for HIE. Although it has certain limitations, the treatment regimen is constantly improving with the continuous improvement in clinical practice [19]. For instance, mild hypothermia therapy can effectively improve the neurological function of children with HIE and inhibit the inflammatory response [20].

In this study, there was no difference in the NBNA score among the three groups on admission. After treatment, the NBNA score increased in all the three groups and was the highest in the combination group, while that in the mild hypothermia group was higher compared with the routine group. It is suggested that mild hypothermia combined with GM1 can better improve the neural function of neonates with HIE, which is consistent with the results of previous research [21]. Mild hypothermia therapy is used for a variety of cerebrovascular diseases such as cerebral hemorrhage and has been proven to protect the brain tissues and reduce intracranial pressure [22], while GM1 for the treatment of HIE has been shown to improve not only the short-term development of nervous system, but also the long-term brain function of neonates. Based on the above research, this study further proved that GM1 combined with mild hypothermia treatment has a better protective efficacy on the neural function of neonates with HIE. The possible mechanism may be that the metabolic rate of brain tissues and cell energy are slowed down under mild hypothermia, which reduces neuron necrosis and apoptosis [23]. While low temperature environment alone cannot restore the damaged nerve cells, GM1, as an essential substance for the regeneration and development of brain nerves, can promote nerve regeneration [24], which makes up for the shortcomings of mild hypothermia therapy. In combination, the two treatments complement each other to achieve better curative effects.

SOD is an active substance derived from living organisms, which can eliminate harmful substances produced during metabolism [25]. It is confirmed that the SOD level in neonates with HIE is significantly lower than that of normal neonates [26]. In this study, the SOD level increased in all three groups after treatment, with the most significant increase in the combination group, suggesting that the combined treatment for HIE can more effectively increase the SOD level in neonates. Research has shown that during the occurrence and development of HIE, the level of SOD in neonates decreases, which further leads to lipid peroxidation and cell damage [27], while hypothermia therapy can protect neurological function in brain damage caused by ischemia and hypoxia by increasing the level of SOD. Another study also showed that GM1 combined with mild hypothermia treatment for HIE could reduce oxidative stress by enhancing SOD activity and promoting the recovery of neural function in neonates [28]. The results of this study are consistent with the above studies, which further proves that mild hypothermia combined with GM1 can increase SOD activity and protect brain function in neonates with HIE.

NSE and S-100*β* protein are widely present in neurons and are released into the blood and cerebrospinal fluid in large quantities when the brain tissue is damaged. Therefore, the degree of neuronal damage can be inferred based on the serum NSE level. In addition, NSE has been proven to have a certain effect on predicting future neurodevelopmental outcome in neonates with HIE [29]. S100*β* protein can inhibit neuronal repair and accelerate neuronal cell apoptosis after brain injury. In this study, NSE and S100*β* protein decreased in all the 3 groups after treatment, with most significant decreases in the combination group, indicating that GM1 combined with mild hypothermia treatment for HIE can better avoid neuronal damage in neonates, which is consistent with the results of previous studies [30]. Possible reasons could be that mild hypothermia therapy can help restore the neural function of patients with brain injury and reduce brain damage, and that GM1 can cause intracellular calcium overload and reduce brain edema in neonates with HIE. Therefore, in combination, the two further reduced the brain damage in neonates with HIE.

Plasma NPY is widely distributed in the central nervous system, showing strong vasoconstrictor effect. The damage of the nervous system in neonates with HIE leads to the release of NPY into the blood, which inhibits vasodilators and hinders brain development in neonates. It is shown that the plasma NPY level in neonates with HIE is positively correlated with the severity of HIE [31]. In this study, the level of NPY decreased in all the 3 groups after treatment, with the lowest level observed in the combination group, demonstrating that mild hypothermia combined with GM1 can better reduce the impact of HIE on the brain development of neonates. Possible reasons could be that the low temperature environment can reduce the demand for oxygen and energy of brain cells, and that GM1 can improve cerebral blood flow dynamics in neonates with HIE. Therefore, the two work together to alleviate the cerebral ischemia and hypoxia and reduce the damage to brain function in neonates with HIE [32].

This study found that neonates in the combination group had the shortest recovery time for clinical signs, the highest total effective rate, and the least number of complications. Epilepsy and cerebral palsy are common complications of HIE, and their inducement is related to permanent damage of central nervous system caused by HIE. In addition, routine hypothermia therapy for HIE children also presents a risk of respiratory failure, which may be associated with oxygen limitation due to hypoxic ischemic events [33, 34]. The data of this study confirmed that mild hypothermia therapy combined with GM1 can not only improve the treatment effectiveness of HIE but also reduce the risk of epilepsy, cerebral palsy, and respiratory failure.

The novelty of this study lies in the analysis of the clinical advantages of mild hypothermia therapy combined with GM1 in the treatment of neonatal asphyxia complicated by HIE from the aspects of neurological function recovery, biochemical indicators, clinical signs recovery, efficacy, and complications, which can provide clinical basis for the treatment of the disease, optimize the treatment options, and improve the treatment efficacy and safety, whereas limited by conditions, this study has some deficiencies. First, the specific efficacy of mild hypothermia therapy combined with GM1 on neonates with different degrees of HIE was not observed. Second, there was no follow-up observation on the long-term intelligence level of the three groups of neonates. Therefore, in future studies, the sample should be expanded and the observation time span should be extended for further in-depth research.

In summary, the combination of hypothermia therapy and GM1 for the treatment of neonatal asphyxia complicated by HIE can improve the neural function and the recovery of clinical signs in neonates, with high efficiency and few complications, which is worthy of clinical application.

## Figures and Tables

**Figure 1:** Comparison of neural function among the three groups before and after treatment. Compared with that at admission, ^∗^*P* < 0.05 and ^∗∗∗^*P* < 0.001; compared with the routine group, ^###^*P* < 0.001; compared with the mild hypothermia group, ^&^*P* < 0.05. GM1: monosialotetrahexosylganglioside.

**Figure 2:** Comparison of levels of SOD, NPY, S-100*β*, and NSE before and after treatment among the three groups. (a) Comparison of SOD levels before and after treatment among the three groups; (b) comparison of NPY levels before and after treatment among the three groups; (c) comparison of S-100*β* levels before and after treatment among the three groups; (d) comparison of NSE levels before and after treatment among the three groups. Compared with that at admission, ^∗^*P* < 0.05 and ^∗∗∗^*P* < 0.001; compared with the routine group, ^###^*P* < 0.001; compared with the mild hypothermia group, ^&^*P* < 0.05. GM1: monosialotetrahexosylganglioside; SOD: plasma superoxide dismutase; NPY: neuropeptide Y; NSE: neuron-specific enolase.

**Figure 3:** Comparison of the recovery of clinical signs among the three groups during treatment. Compared with the routine group, ^###^*P* < 0.001; compared with the mild hypothermia group, ^&^*P* < 0.05. GM1: monosialotetrahexosylganglioside.

**Table 1:** Comparison of general data among the three groups (*n*, *x̅*±sd).

Item	Routine group	Mild hypothermia group	Combination group	*χ* ^2^/*F*/*t*	*P*
Sex (male/female)	18/12	17/13	14/16	1.165	0.559
Gestational age (weeks)	37.4 ± 2.1	36.9 ± 1.9	37.6 ± 2.0	0.973	0.382
Day age (days)	1.1 ± 1.1	1.2 ± 1.1	1.2 ± 1.0	0.088	0.916
Birth weight (kg)	3.0 ± 0.5	3.1 ± 0.6	3.0 ± 0.6	0.309	0.735
Asphyxia score	11.4 ± 1.4	11.2 ± 1.5	10.9 ± 1.1	1.052	0.354
5 m Apgar score	4.2 ± 1.2	3.9 ± 1.1	3.9 ± 1.3	0.622	0.539
HIE severity (mild/moderate/severe, *n*)	10/18/2	8/17/5	7/15/8	4.440	0.350

Note: HIE: hypoxic ischemic encephalopathy.

**Table 2:** Comparison of neural function among the three groups before and after treatment (*x̅*±sd).

Group	Number of cases (*n*)	NBNA score on admission	NBNA score after treatment
Routine group	30	29.20 ± 3.21	31.17 ± 3.38^∗^
Mild hypothermia group	30	28.39 ± 3.46	34.42 ± 3.57^∗∗∗^^###^
Combination group	30	28.96 ± 3.01	36.57 ± 3.15^∗∗∗^^###&^

Note: Compared with that at admission, ^∗^*P* < 0.05 and ^∗∗∗^*P* < 0.001; compared with the routine group, ^###^*P* < 0.001; compared with the mild hypothermia group, ^&^*P* < 0.05. NBNA: neonatal behavioral neurological assessment.

**Table 3:** Comparison of SOD, NPY, S-100*β*, and NSE levels among the three groups before and after treatment (*x̅*±sd).

Group (*n*)	Time	SOD (U/ml)	NPY (ng/L)	S-100*β* (ng/ml)	NSE (U/ml)
Routine group (*n* = 30)	On admission	110.57 ± 15.32	152.56 ± 3.18	5.68 ± 1.32	15.04 ± 1.59
	After treatment	118.85 ± 16.28^∗^	150.56 ± 3.28^∗^	4.94 ± 1.45^∗^	13.92 ± 1.73^∗^
Mild hypothermia group (*n* = 30)	On admission	112.34 ± 14.89	152.84 ± 3.52	5.52 ± 1.31	15.12 ± 1.38
	After treatment	132.50 ± 15.11^∗∗∗^^###^	142.33 ± 2.78^∗∗∗^^###^	3.65 ± 1.43^∗∗∗^^###^	10.82 ± 1.68^∗∗∗^^###^
Combination group (*n* = 30)	On admission	113.56 ± 16.82	153.79 ± 3.14	5.64 ± 1.38	15.35 ± 1.46
	After treatment	141.78 ± 16.92^∗∗∗^^###&^	140.58 ± 2.81^∗∗∗^^###&^	2.92 ± 1.21^∗∗∗^^###&^	9.82 ± 1.84^∗∗∗^^###&^

Note: Compared with that at admission, ^∗^*P* < 0.05 and ^∗∗∗^*P* < 0.001; compared with the routine group, ^###^*P* < 0.001; compared with the mild hypothermia group, ^&^*P* < 0.05. SOD: plasma superoxide dismutase; NPY: neuropeptide Y; NSE: neuron-specific enolase.

**Table 4:** Comparison of the recovery of clinical signs among the three groups during treatment (*x̅*±sd).

Group (*n*)	Consciousness recovery time (d)	Reflex recovery time (d)	Muscle tension recovery time (d)
Routine group (*n* = 30)	6.74 ± 1.77	6.98 ± 1.38	6.68 ± 1.29
Mild hypothermia group (*n* = 30)	5.15 ± 1.65^###^	5.52 ± 1.57^###^	5.41 ± 1.23^###^
Combination group (*n* = 30)	4.28 ± 1.48^###&^	4.69 ± 1.61^###&^	4.57 ± 1.42^###&^

Note: Compared with the routine group, ^###^*P* < 0.001; compared with the mild hypothermia group, ^&^*P* < 0.05.

**Table 5:** Comparison of efficacy among the three groups (*n*, %).

Group (*n*)	Markedly effective	Effective	Ineffective	Total effective rate	*χ* ^2^	*P*
Routine group (*n* = 30)	4 (13.33)	14 (46.67)	12 (40.00)	18 (60.00)	15.792	<0.001
Mild hypothermia group (*n* = 30)	12 (40.00)	12 (40.00)	6 (20.00)	24 (80.00)		
Combination group (*n* = 30)	18 (60.00)	9 (30.00)	3 (10.00)	27 (90.00)		

**Table 6:** Comparison of complications among the three groups during treatment (*n*, %).

Group (*n*)	Epilepsy	Cerebral palsy	Respiratory failure	Total incidence	*χ* ^2^	*P*
Routine group (*n* = 30)	9 (30.00)	5 (16.67)	1 (3.33)	15 (50.00)		
Mild hypothermia group (*n* = 30)	8 (26.67)	4 (13.33)	0 (0.00)	12 (40.00)	13.026	0.043
Combination group (*n* = 30)	2 (6.67)	1 (3.33)	0 (0.00)	3 (10.00)		

## Data Availability

The labeled dataset used to support the findings of this study are available from the corresponding author upon request.
